This article has been retracted.

# Surgical Treatment of Hand and Foot Gout Stone and Influence Factors on Prognosis

**DOI:** 10.1155/2022/4877708

**Published:** 2022-09-26

**Authors:** Xudong Qiu, Bo Zhao, Xingxu Du, Shuo Jin, Weiyan Zhao

**Affiliations:** ^1^Department of Hand Surgery, The Affiliated Hospital of Beihua University, Jilin, Jilin 132011, China; ^2^Department of Endocrine, The Affiliated Hospital of Beihua University, Jilin, Jilin 132011, China

## Abstract

**Purpose:**

To explore the technique of surgical treatment of hand and foot gout stone by using 3D CT reconstruction images and influence factors on prognosis.

**Method:**

48 cases of hand and foot gout were treated surgically and retrospective analyzed. Before operation, we used 3D CT reconstruction images to check the accurate site and amount of uric acid (white chalk foam) deposition. Different surgical methods were applied depending on the different deposition site of urine acid stone. The frequency of gout attack and blood uric acid was compared before and after surgery. Patients were followed up to observe the recovery and recurrence and then analyzed the reason of unsuccessful healing.

**Result:**

Sutures were removed 2 weeks after operation in all cases. The frequency of gout attack and blood uric acid of patients 3 months after operation was lower than those before operation, and the differences were statistically significant. Follow-up ranged from 1 to 3 years, with an average of 1.8 years. Three cases were not followed up. The remaining 45 cases were healed in the first stage. 40 cases had improved joint function, increased range of motion, and relieved discomfort after movement. 5 cases had no improvement in joint function after operation, and 3 of them had gout stone recurrence (nonoperative area) and were treated by second hospital operation.

**Conclusion:**

Surgical treatment of gout stone in hand and foot under the guidance of three-dimensional CT reconstruction image can effectively alleviate the local symptoms of gout stone and improve the function of hand and foot. Deep tissue can be thoroughly washed by the pressure of pulse gun after resection of the lesion, which can reduce the incidence of gout stone. Malnutrition, hypoproteinemia, and residual urine acid in the wound are the main reasons for unsuccessful healing.

## 1. Introduction

Gout is painful inflammation of the joints caused by high uric acid levels and purine metabolism disorders [1–3]. As the standard of living increases, the incidence of gout increases and tends to be younger, closely related to alcohol consumption, and some patients are associated with genetic factors [4, 5]. However, the continuous rise of blood uric acid will lead to the formation of tophite of different sizes when urate crystals precipitate and deposit in tissues or organs, bones, and joints, resulting in local deformity and swelling, pain, redness, ulceration, and dysfunction [6, 7]. Gout stone is a sign of chronic gout and a chronic granulomatous disease, which appears in a few years after the first attack of gout [8]. In some cases, it will affect the appearance of the patients and make them feel inferior [9]. In other cases, it will cause joint stiffness and deformity, even disability, loss of labor ability, and inability to take care of themselves, and seriously affect the quality of life of the patients [10]. Thus, it is crucial to prevent gout stone in patients with gout. Early treatment included dietary regulation and medical acid-expelling drugs [11, 12]. But for some patients with severe local gout stone in late stage, surgical intervention is often needed [13]. Because gout stone often occurs all over the body, and the joint of hands and feet is common, it often causes swelling of the whole joint and restriction of movement.

At present, three-dimensional CT reconstruction can make gout stone lesions appear green, distinguish from normal bone, and define the model of the lesion [14, 15]. Before the advent of advanced imaging technology, the understanding of gout pathology was mainly based on the optical microscopy of gout stone and periarticular bone, supplemented by plain radiography to determine the X-ray morphology and distribution of erosion [16]. However, this method tends to investigate severe erosive gouty arthropathy. Specimens used for histopathology are usually from amputated fingers or limbs. Chronic excretion of gout stone is often a secondary infection [17]. Helical multislice CT scanning was seen to be a potential role in the diagnosis of gout, mainly because it can obtain very high-resolution three-dimensional images to describe gout stone [18]. The density of gout stone is usually 160-170 Hounsfield units, which is expressively different from the density of soft tissue and bone [19]. Helical CT scan also has the advantage of imaging a larger area than most MRI scans, so it can describe the pattern of joint involvement [20].

Thus, combined with three-dimensional CT images, we can accurately remove the lesions of gout stones in hands and feet and reduce tissue damage. Especially for deep incision gout stones, it is not easy to omit, so as to reduce the recurrence rate of surgical area. However, there have been few reports on the surgical records of patients with gout stone, thus, the novelty and motivation of this study are to comprehensively analyze the surgical treatment techniques and prognostic factors of gout stone by combining 3D CT images and surgical experience, so as to provide reference for subsequent clinical treatment of gout stone. Herein, since 2013, we have treated 48 cases of gout stones in hands and feet clinically. Now, we summarize as follows.

## 2. Materials and Methods

### 2.1. General Information

48 cases, all male, aged 19-79 years, average age 51 years; course of disease (1-25 years, average 12.1 years); site of disease: multiple nodules in hand-foot joint and subcutaneous part, including 4 cases of gout in wrist joint, accompanied with carpal tunnel syndrome [21]. This study was approved by the hospital ethics committee. Informed consent was obtained from the patients and their families, and the informed consent was signed. Inclusion and exclusion criteria: patients with at least one follow-up visit between 1 January 2013 and 31 December 2021 were included in the present analysis. Patients with complete clinical information and imaging data were included. Patients in whom gout was associated with a haematological malignancy or other malignant disease not confirmed to be in remission were excluded.

### 2.2. Clinical Manifestations

It is mainly manifested in four aspects:

1. Gouty stones invade skin and subcutaneous tissues only. They are isolated gouty stones and do not invade deep tendinous tissues and joints
2. Gouty stones invade tendons or joints and ligaments, showing swelling of fingers or toes, swelling of joints, and limited movement
3. Gouty stones invade bone, manifested as finger (phalange) destruction, incomplete articular surface, limited joint movement, and obvious hand deformity
4. Gout stone is combined with peripheral nerve compression, and the most common part is the wrist. Gout deposits form on the surface of tendons or ligaments in carpal canal, and neurological symptoms appear when gout stone compresses median nerve

48 cases showed multiple subcutaneous gout nodules in hands and feet, joint pain, swelling, and stiffness, and 4 cases had carpal tunnel syndrome. There were 3 cases with abnormal serum uric acid before operation, the highest was 683 *μ*mol/L (normal range: 150-380 *μ*mol/L for males and 100-300 *μ*mol/L for females). All patients were applied X-ray examination of articular position: the articular surface showed worm-like destruction and joint space narrowed; CT three-dimensional reconstruction of hand or foot was performed before operation in all patients, and the reconstructed images showed that the gout area was green imaging, which was significantly different from normal bone (Figure 1).

### 2.3. Therapeutic Methods

Surgical treatment was used in all 48 cases.

#### 2.3.1. Preoperative Preparation

1. Attention should be paid to adjusting diet, controlling the intake of high purine diet, maintaining urine volume of more than 2 500 ml per day, taking alkaline food or drugs to alkalize urine. Urine pH value should be controlled to about 6.5
2. Give probenecid or allopurinol orally to control the level of serum uric acid

The range of operation was determined by marking the area of uric acid deposition in CT images and the symptoms and signs of patients before operation.

#### 2.3.2. Surgical Methods

Brachial plexus or epidural nerve block anaesthesia was used. A large amount of uric acid (white chalk foam) deposited in subcutaneous soft tissue, tendon, articular capsule, or bone invasion was found in the green CT image area during operation (Figure 2). For the isolated gout stone in the subcutaneous soft tissue can be completely removed. For gout stone invading joints and tendons, part of flexor digitorum superficialis tendon and joint capsule shall be removed to ensure that uric acid crystals are completely removed, and the hand function shall be preserved as much as possible. For the gout stone invading the bone, the gout stone injury in cartilage and cancellous bone shall be completely removed, and the severely damaged interphalangeal joint shall be fixed by joint fusion. For fingers (toes) that are almost completely eroded by uric acid, consider cutting off the fingers (toes). When the finger is almost completely eroded by uric acid, finger amputation (toe) can be considered; carpal tunnel incision, lesion excision, and neurolysis are performed in patients with carpal tunnel syndrome; after gout stone excision, a large number of salines is used to wash the wound repeatedly, and the residual uric acid can be thoroughly washed out by the pressure of the pulse gun. The incision suture was removed 14 days after operation.

#### 2.3.3. Postoperative Management

1. Monitor the changes of serum uric acid, and continue to maintain the preoperative treatment, so as to control the serum uric acid in normal level. Colchicine can be administered orally for 3 to 5 days if acute gout attack occurs
2. Two weeks after operation, it is suggested that the operation area be immobilized to promote wound healing
3. Early rehabilitation physiotherapy, assisting patients with joint function exercise, as soon as possible to restore limb and joint function

### 2.4. Indicator for Further Observation

1. Compare the frequency of gout attack 3 months after surgery
2. Compare the blood uric acid level 3 months after surgery: 5 mL fasting venous blood was extracted and centrifuged at 3000 r/min for 15 min, serum was obtained to detected the blood uric acid level using ELISA assay, and the kits were purchased from Shanghai Junrui Biotechnology Co., Ltd.
3. Long-term follow-up after surgery to observe the cure of patients (completely dissolved monosodium urate crystals, all crystals removed surgically and no new crystals formed afterwards), statistics of recurrence. Access the patients' joint function, the range of motion. Record the discomfort after movement

### 2.5. Statistical Analysis

SPSS22.0 software (IBM, Chicago, IL) was used for data processing to represent measurement data, paired *t* test was used between groups, counting data was expressed as percentage, *P* < 0.05 was considered statistically significant.

## 3. Result

### 3.1. Gout Attack Frequency and Blood Uric Acid Level

The frequency of gout attack and blood uric acid of patients 3 months after operation were lower than those before operation, and the differences that were statistically significant (*P* < 0.05) are shown in Table 1.

### 3.2. Follow-Up Results

Postoperative follow-up 1 ~ 3 years, an average of 1.8 years. 3 cases were not followed up. The remaining 45 cases were healed in the first stage. 40 cases had improved joint function, increased range of motion, and relieved discomfort after movement. 5 cases had no improvement in joint function after operation, and 3 of them had gout stone recurrence (nonoperative area) and were treated by second hospital operation. 2 cases with special gout were shown in Figures 3 and 4.

## 4. Discussion

Gout is a metabolic disorder in internal medicine. Urate deposition in the body can cause the destruction of hand and foot joint ligaments and soft tissues [22]. Surgical removal of gout stones can reduce the total amount of uric acid in the body, slow down the progress of lesions, and prevent irreversible damage caused by bone, joint, tendon, and nerve invasion [23]. In addition, gout stone is a huge reservoir of gout stones, which can continuously release uric acid to the blood [24]. Urate deposits in the renal interstitium and tubules to form kidney stones [25], so surgical removal of some gout stones can reduce the burden of the kidney and protect the kidney. With the help of three-dimensional CT image operation, the scope of operation can be cleared more clearly, the deep hidden uric acid can be thoroughly removed, the residual uric acid can be reduced, the side-effects can be avoided, and the recurrence can be effectively prevented.

### 4.1. Surgical Indications of Gout Stone in Hand and Foot

1. Hand and foot gout stones protruding the skin surface or swelling obvious, affecting the shape
2. Invading the tendon or joints, affecting hand and foot activity and functional disorders
3. Gout stone combined with nerve compression symptoms such as sensory numbness and dyskinesia
4. Local gout stone invasion of the skin, causing breakage or coinfection

### 4.2. Preoperative Localization of Gouty Stones Based on Clinical Manifestations of Patients and CT Reconstructed Images

Gout stones often protrude on the skin surface at the back of the hands and foot, but during the operation, it was found that gout stones also invaded the palmar tissue, sometimes with uric acid deposition around the joint. Because the three-dimensional reconstruction image indicates the three-dimensional image, preoperative three-dimensional CT imaging can show the exact location of urate deposition, especially for patients with palmar lesions and no obvious symptoms, so as to prevent the omission during operation. Because of the frequent occurrence of gout stones, surgical resection is not necessary, so communication with patients before operation is needed to determine the extent of surgical resection. Referring to the three-dimensional CT images, surgical treatment was performed on the sites with obvious urate deposition or local gout nodules on physical examination, which obviously affected the shape and joint activity of hands and foot.

### 4.3. Surgical Characteristics of Gout Stone

Different surgical methods are adopted according to the extent of gout stone invasion.

1. Direct excision of isolated gouty stones with simple invasion of superficial subcutaneous soft tissue
2. Gouty stones involving joints and tendons should be preserved as much as possible, such as ligaments, joint capsules, and tendons of flexor digitorum profundus. Because the essence of gouty stones resection is subtractive surgery, it is impossible to cure them thoroughly, so we should weigh the advantages and disadvantages and not injure important tissues and functions simply for the purpose of thorough removal of gouty stones. Tendons with severe injuries but not major functions such as flexor digitorum superficialis can be resected
3. Some gout stones invade phalanges or metacarpals. The bone marrow cavity is full of gout stones, which cannot be completely removed. Small-scale gout stones can be curettage. If single phalanges or phalanges are severely damaged or articular surface is obviously damaged, focal debridement and joint fusion can be performed
4. Carpal tunnel incision decompression combined with carpal tunnel syndrome, nerve release, and simultaneous removal of gout deposited in carpal tunnel

### 4.4. Precautions of Gout Surgery and the Advantages of Pulse Gun Therapy

First of all, the design of incision is very important, pay attention to protecting the blood supply of the skin margin, separating as sharply as possible during the operation to prevent skin necrosis; the affected tissues (such as nerves, tendons, blood vessels, and ligaments) cannot be completely removed during the operation; otherwise, the function of the hand will be lost; after the removal of the lesion, the surgical area needs to be soaked and washed with a large amount of sodium chloride to reduce the deposition of uric acid in the lesion area. After excision of the lesion, we use the pulse gun to wash the lesion thoroughly and reduce the recurrence rate by removing the residual uric acid in the soft tissue by vibration and suction under negative pressure.

### 4.5. Preoperative Treatment of Gout Stone

Comprehensive medical treatment must be supplemented before operation, and the patient's general condition should be carefully evaluated. Because gout patients are often accompanied by hypertension, diabetes mellitus, hyperlipidemia, coronary heart disease, kidney stones, renal insufficiency, and so on, it is necessary to comprehensively evaluate the patient's ability to withstand surgery and pay attention to the treatment of complications to prevent the occurrence of intraoperative accidents and nonhealing of wounds after surgery and not reluctantly operate. At the same time, the level of serum uric acid should be kept at a relatively low level, because during the removal of gout stones and uric acid crystals during operation, some uric acid crystals will dissolve and absorb into the blood, which will easily lead to acute gout attack after operation [26]. After operation, attention should be paid to monitoring biochemical indicators and changes in renal function, and attention should be paid to adjusting the level of serum uric acid to normal range. In order to promote wound healing, attention should be paid to limb immobilization, protein supplementation, and local physiotherapy to improve circulation within 2 weeks after operation. If the patient is old age, poor nutritional status, cardiopulmonary function, and renal function insufficiency do not consider the surgical treatment.

### 4.6. Selection of Operative Time for Gout Stone Surgery

At present, the clinical consensus is that gout stone surgery is the best treatment, but the timing of surgery is still controversial. Some scholars believe that some gout stones can be eliminated by drug treatment or self-elimination. Only when gout stones cause dysfunction and other complications, they need to be removed surgically [27]. Others believe that gout stones are equivalent to a uric acid storage bank, which continuously releases uric acid into the blood, leading to the acute onset of gout [28]. Early surgical excision can not only reduce the storage of uric acid in vivo, reduce the level of uric acid in peripheral blood, and reduce the burden of excretion of uric acid in kidney, but also prevent gout stone from further erosion and destruction of bone, joint, tendon, nerve, blood vessel, and other important tissues and organs, prevent skin ulceration, preserve and restore hand function, and improve the appearance. Therefore, it is advocated that once gout stone is removed, it can improve the appearance. It was found that early surgical resection should be performed. Some gout patients may have normal serum uric acid, but the local symptoms are obvious.

Therefore, three-dimensional CT reconstruction is not only a diagnostic indicator of gout but also can monitor the progress of gout, and early surgery when symptoms occur. Especially gouty stones near joints and ligaments should be removed as early as possible; otherwise, the whole joint and cartilage will be eroded by gouty stones gradually, and joint function will be lost.

### 4.7. The Reasons for Unsuccessful Healing

Anemia, hypoprotenemia, residual urinate acid in the wound, or excessive incision in one operation can cause the unsuccessful healing after operation. So we should give enough preparation about health and nutrition before operation to recover anemia and hypotenemia. And we cannot resolve all of the problems for the patient with gouts more than 8 cites in one person at one operation. Moreover, studies have shown that by lowering serum urate levels at least below 6 mg/dl (360 *μ*ml/L), dissolution of the pathogenic monosodium urate crystals is achieved, and disappearance of clinical features of gout can be obtained [29, 30].

## 5. Conclusion

In conclusion, preoperative CT three-dimensional reconstruction can identify the lesions of gout stones in hands and feet, make the operation more targeted, reduce the omission of lesions and side injuries, and pay attention to reduce the removal of nerves, tendons, blood vessels, ligaments, joint capsules, and other important tissues during the operation, so as to maximize the preservation of hand function. High frequency pulsed flushing with pulse gun can thoroughly flush the residual uric acid in the lesion area, which can make the operation achieve satisfactory results. However, in order to control the recurrence of gout stones and the onset of gout, it is necessary to combine dietary therapy with the application of hypo uric acid drugs, which can be combined with inhibiting the formation of uric acid and persisting in systematic and comprehensive treatment for a long time. Recently, it has been reported that uricase drugs have the effect of dissolving uric acid. At the same time, three-dimensional CT was reviewed regularly to monitor the progress of patients.

The presented study still have limitations, the follow-up of the patients should include relative biochemical indicator. Reducing sUA levels to target is the main strategic concept to “cure” gout [31]. At present, the ideal way to treat gout stone is to locate it by three-dimensional CT imaging, inject a specific enzyme into the lesion area to dissolve uric acid stone, and then remove gout stone under arthroscopy, which is also the direction of our future research.

## Figures and Tables

**Figure 1:** Preoperative three-dimensional CT reconstruction shows green areas of gout stone deposition.

**Figure 2:** The lesion area of the left hand in the operation is consistent with the preoperative CT image.

**Figure 3:** The lesion area of the right hand in the operation. (a) The toph invaded the superficial flexor digitorum tendon and pressed the median nerve in the carpal canal. (b) The superficial flexor digitorum tendon resection, toph removal, and median nerve release were performed.

**Figure 4:** The lesion area of the left foot in the operation. (a) Topout stone encroached sole middle phalanx of the little toe of the foot. (b) Middle phalanx resection was performed. (c) Arthrodesis was performed.

**Table 1:** Gout attack frequency and blood uric acid level.

Time point	The frequency of gout attack (times/month)	Blood uric acid level (*μ*mol/L)
Before surgery (*n* = 48)	2.71 ± 0.46	585.66 ± 34.41
3 months after surgery (*n* = 48)	0.90 ± 0.42	333.13 ± 25.23
*t*	20.1318	41.0040
*P*	<0.0001	<0.0001

## Data Availability

The labeled dataset used to support the findings of this study are available from the corresponding author upon request.
